# Multi-sensor information fusion detection system for fire robot through back propagation neural network

**DOI:** 10.1371/journal.pone.0236482

**Published:** 2020-07-24

**Authors:** JunJie Zhang, ZiYang Ye, KaiFeng Li

**Affiliations:** School of Electronic and Electrical Engineering, University of Leeds, Leeds, United Kingdom; University College London, UNITED KINGDOM

## Abstract

**Objective:**

To reduce the danger for firefighters and ensure the safety of firefighters as much as possible, based on the back propagation neural network (BPNN) the fire sensor multi-sensor information fusion detection system is investigated.

**Method:**

According to previous studies, the information sources and information processing methods for the design of this study are first explained. Then, the basic structure and flowchart of the research object in this study are designed. Based on the structure diagram and flowchart, the BPNN is selected to fuse the feature layers in this study, and the fuzzy control is selected to fuse the decision layers in this study. The multi-sensor information fusion detection system collects information for the sensors first, processes the collected information, and sends it to the processor of the robot. The processor analyzes and processes the received signal, and transmits the obtained information to the control terminal through the wireless communication system.

**Results:**

Through the tests in this study, it is found that when the number of hidden layer nodes of the BPNN is 7, the optimal training result is obtained. On this basis, the test of BPNN in this study is performed. The test results show that after 127 iterations, the error of the BPNN reaches the lowest target value, indicating that the BPNN achieves an excellent level of accuracy. The trained BPNN has a running time of 0.0276 s and a mean square error of 0.0013. The smaller the mean square error value is, the higher the accuracy of the BPNN is, which shows that the BPNN meets the high precision requirements of this study.

**Conclusion:**

The research on the multi-sensor information fusion detection system of fire robots in this study can provide theoretical support for the research on forest fire detection in China. Since the proposed BPNN-based robot is applied to the inspection and processing of forest remaining fire, the results are applicable to the forests of various countries, with a wide range of applications.

## 1. Introduction

This year, the world has experienced frequent fires. Major forest fires in Sichuan Province in China, tropical rain forest fires in Brazil, and continuous fires in Australia have caused immeasurable losses to humans. A large number of animals have been burned to deaths, while the survived animals have also lost their homes [1, 2]. Fire is a natural disaster that is difficult to predict, and the harm caused by the fire is also difficult to estimate, especially forest fires. Forest fires are often difficult to extinguish all sources of disaster. Many forest fires are secondary fires caused by incomplete fires. Because of the complex forest environment, flames are easily covered by vegetation such as weeds. Therefore, it is difficult to completely extinguish the fire [3]. At present, most clean up works of remaining fires are undertaken by firefighters. In the jungle with a complex environment, the safety of firefighters is difficult to guarantee. The fires may spread again in the forest at any time, and it is difficult for firefighters to inspect the remaining fires in time and extinguish these fires, resulting in greater losses [4]. Although fire detection technology is available to assist firefighters in the search and rescue of fire spots, the traditional detection technology is not ideal for the detection of remaining fires. Therefore, despite the great efforts of people all over the world, fires events still cannot be effectively prevented.

With the development of robotics in recent years, researchers have begun to look for a new method, which is to clean up the fire remaining fire by robots. Robots find forest fires more efficiently and quickly and greatly reduce firefighters’ pressure for extinguishing the fire. Mizuno et al. (2019) researched a fire robot system composed of multiple autonomous robots, proposed a robot path planner, applied the path planner to an actual robot, verified whether the generated path was suitable for a fire robot system, and finally proved that the proposed planner had wide applicability [5]. Rao et al. (2019) combined the intelligent water droplet algorithm with the differential evolution algorithm to study the fire bird robot. The simulation results showed that the method could guide the robot to predict the nature of obstacles and generate optimal and safe motion tracks in a dynamic workspace [6]. Sowah et al. (2016) studied a multi-sensor fire detection system based on fuzzy logic and a web-based notification system. Their research showed that the proposed method had significantly improved the form of timely detection, alarm, and response [7]. Jiang et al. (2017) studied the optimization of dynamic task assignment in fire robot systems and proposed a Pareto-improved secondary task assignment algorithm based on the initial task assignment of the contract network. The results showed that compared with the reinforcement learning algorithm and the ant colony algorithm, the fire fighting time of the designed algorithm was reduced by 26.18% and 37.04%, respectively [8]. Zhang et al. (2014) designed an intelligent fire extinguishing robot to automatically extinguish a fire in a simulated room. The design based on the embedded chip STM32F103 used the sensor group to obtain environmental signals and thereby control the actions of the robot. The intelligent robot could automatically track the path, avoid obstacles, find the source of the fire, extinguish the fire accurately and quickly, and finally return to the origin. The experimental results showed that the intelligent robot could run flexibly and quickly, and had the characteristics of high accuracy and easy operation [9]. According to previous research results, it is found that there are a large number of fire detection studies, and the methods are pretty mature.

However, the research on forest remaining fires is more complex, and related research is scarce. Therefore, this study explores the detection methods of forest remaining fires based on the back propagation neural network (BPNN). According to previous studies, the information sources and information processing methods for the design of this study are first explained. Then, the basic structure and flowchart of the research object in this study are designed. Based on the structure diagram and flowchart, the BPNN is selected to fuse the feature layers in this study, and the fuzzy control is selected to fuse the decision layers in this study. The innovation of this study lies in the utilization of robots to complete the entire forest remaining fires detection process, which greatly reduces labor costs and ensures the maximum safety of firefighters. It is hoped that the investigation of forest fire detection robots can contribute to the detection of forest fires in various countries and minimize the damage to personnel.

## 2. Method

### 2.1 Detection module of forest remaining fires

The process of a fire is very complicated and extremely susceptible to interference from the surrounding environment. Because a series of fire products such as smoke, heat, light, and combustion sounds are generated during the fire, the fire detection method also extends from these aspects to flame sensor detection, image sensor detection, temperature sensor detection, and gas sensor detection. In a variety of ways, such as using sensors to separate the characteristic information from the fire, the purpose of identifying the fire is achieved [10, 11].

In addition, the way to choose the information to be researched among much environmental information is a very important link. Too little information will cause too much interference, which is difficult to distinguish; meanwhile, too much information will cause a long calculation process, making it fail to achieve rapid fire detection. Under normal circumstances, the content of carbon monoxide in the air is low. In the event of a fire, carbon monoxide will be released in large quantities due to combustion; therefore, the content of carbon monoxide in the air will be an indicator of fire detection. Also, the most obvious detection indicators of fires are the increase in temperature, the increase in smoke concentration, and the enhancement of infrared signals. Therefore, this study uses temperature, infrared signal strength, smoke concentration, and carbon monoxide concentration as the detection parameters of the system to form the information source of the sensor fusion system.

The temperature sensor selected for this study is the DS18B20 digital temperature sensor. This temperature sensor has the advantages of being easy to use and does not require analog-to-digital conversion. The working voltage of the temperature sensor is 3–5.5 V, and the temperature measurement range is -55-125°C, with an accuracy ± 0.5°C. The smoke sensor is gas-sensitive smoke sensor MQ-2, and the carbon monoxide gas sensor is board-load MQ-7.

The other major link to the fire detection process is the intelligent processing algorithm in fire detection. The signals detected by the sensors cannot directly predict when will a fire occurs, and these signals are often mixed with other interference signals. Therefore, it is difficult to distinguish them, and the detection of the collected signals is one of the most important issues in fire detection [12]. Due to the high false alarm rate and missed alarm rate of traditional fire detection algorithms, people have developed various algorithms for fire detection. At present, the algorithms used in fire detection mainly include artificial neural networks (ANN), fuzzy processing, and the combination of both. The fire detection algorithms combined with ANN and fuzzy processing make up for each other’s shortcomings in the process of utilization, thereby achieving a better fire detection effect [13]. Therefore, the fire detection algorithm used in this study is a fire detection algorithm combining ANN and fuzzy algorithms.

### 2.2 Fire signal preprocessing

The process of fire occurrence in remaining fires is often a dynamic process. With the continuous change of parameters, the temperature rises and the smoke concentration rises. Therefore, in the process of fire information detection, the original information detected by the sensor must be processed first, such as amplifying, filtering, and analog-to-digital conversion of signals, i.e., processing the detected signals into signals that can be used directly by the fire detection system.

### 2.3 Obstacle avoidance module of the fire robot

The obstacle avoidance function of the fire robot mainly relies on the distance sensor to transmit the position information of the robot. At present, there are various distance sensors on the market, such as ultrasound-based, infrared-based, and laser-based distance sensors [14]. It is very difficult to find suitable sensors for obstacle avoidance of firefighting robots. Laser ranging has high accuracy but its cost is high and it is not suitable for large-scale applications. Infrared-based distance detectors have lower requirements on the environment and better directivity, which also responds quickly to the surrounding environment; however, its short detection distance is more suitable for emergency obstacle avoidance of robots. The ultrasonic-based distance detectors have higher requirements on the environment and it is easy to generate a blind spot when they are close to the object.

Therefore, based on the above analysis, the distance sensors used in the obstacle avoidance of the robot selected in this study are KS103 ultrasonic distance sensor and GP2D12PSD infrared distance sensor.

### 2.4 Fire robot environmental monitoring module

The environmental monitoring module is to observe the current environment of the robot through images and take the current real-time photos. The image collection uses the MV-3000UC color charge-coupled device camera and image grabber. This device is used to photograph the current environment of the robot, and the captured images are transmitted to the control terminal in real-time through the wireless communication device so that the staff can inspect the status of the scene at any time to make the best rescue decisions. The utilization of cameras for real-time photographing greatly reduces manpower expenditures, prevents firefighters from being placed in an extremely dangerous state, and greatly improves the detection efficiency of forest remaining fires.

### 2.5 The whole system of fire robot

The major content of designing the multi-sensor information fusion detection system of the fire robot is the design of the sensor circuit and the controller circuit. The main design idea is that various sensors first collect information, process the collected information, and send the processed information to the robot processor. The processor analyzes and processes the received signals, and transmits the obtained information to the control end through the wireless communication system. The overall system design is shown in Fig 1.

**Fig 1:** System overall design.

The flowchart of the detection system for forest remaining fires is shown in Fig 2.

**Fig 2:** Flowchart of the detection system for forest remaining fires.

As shown in Fig 2, each sensor sends the received information to the robot processor, and the processor processes and analyzes the received information. After analysis, if the result is remaining fires, an alarm is sent to the remote-control end. After the alarm is issued, the fire robot immediately executes the fire extinguishing action. If the fire extinguishing action is not performed, it enters the continuous alarm state. After the system extinguishes the fire, the system continues to enter the state of continuously monitoring remaining fires for efficient remaining fire detection.

The flowchart of the robot’s obstacle avoidance module system is shown in Fig 3.

**Fig 3:** Flowchart of the robot obstacle avoidance module system.

As shown in Fig 3, after receiving the information from the infrared distance sensor and the ultrasonic distance sensor, the robot processes and analyzes the information. If the analysis result shows that there are obstacles, it will actively avoid obstacles. If the obtained detection results show that there are no obstacles, the detection will be continued. After the obstacle avoidance is over, the detection state will be automatically entered to ensure that the robot is in the process of continuous obstacle detection.

### 2.6 Feature layer fusion based on BPNN

In this study, the BPNN method is used for the feature layer-based fusion design. The feature layer has a total of four inputs.

The difficulty of feature layer fusion based on BPNN lies in the design of the number of nodes in the hidden layer. Currently, there is no consistent method for selecting the number of nodes in the hidden layer. However, the selection of this node will be related to the normal operation of the entire network. Therefore, the selection of hidden layer nodes is crucial [15]. In the selection of hidden layer nodes, the principle of “appropriate amount” should be followed. If too many hidden layer nodes are selected, the BPNN will spend too much time on learning, but it may not achieve the best learning results. If too few hidden layer codes are selected, the structure of the BPNN will be too simple to meet the requirements of better recognition, better robustness, and better anti-interference ability of the BPNN proposed in this study [16]. Therefore, based on previous studies, this study determines the number of hidden layers by the following equation.

$$N_{h}=\sqrt{N_{1}+N_{0}}+L$$ (1)

Where: N_h_ is the number of hidden layer nodes sought; N_1_ is the number of input nodes; N_0_ is the number of output nodes; L is an integer between 1 and 10. According to actual training experience, this integer is generally chosen to be a large value, which should generally be greater than half of the sum of the input and output.

The three situations that need to be identified include open flame probability Y1, smoldering fire probability Y2, and interference signal probability Y3. The BPNN feature layer fusion system designed in this study has three layers of input, hidden, and output layers. The neuron nodes are 4, 7, and 3, respectively. The method of selecting the learning step in this study is a dynamic method, i.e., the value of the learning step selected at the training place is large, and the size of the learning step is gradually reduced during the training process. Because the BPNN used in this study is simpler, the step size selection in this study should be between 0 and 1.

### 2.7 Decision layer fusion based on fuzzy control

The major function of the decision-making layer is to analyze the output value of the BPNN to obtain a certain result. Since the feature layer gives a probability value, the decision-making layer needs to comprehensively analyze the probability value to obtain a certain result [17].

The main processes of fuzzy control are precise fuzzy, the establishment of fuzzy rules, fuzzy reasoning, defuzzification, and generation of input and output rule tables. Precise fuzzy is to describe precise numerical values in life as vague language such as “large, medium, and small”. Also, adjective vocabulary can be added to refine it as needed. After performing a precise amount of fuzzification, fuzzy rules need to be determined, i.e., rules that can be described in language are extracted based on daily experience and intuition. Fuzzy rules need to have complete, reasonable, and consistent characteristics, which can improve the efficiency of the fuzzy control process [18].

The fuzzy inference method used in this study is the most commonly used arithmetic method of Madani fuzzy implication in fuzzy inference [19,20]. After the fuzzy reasoning is completed, the reasoning result needs to be embodied in a specific description. This study uses the maximum membership method to perform defuzzification to generate the input and output rules required by this study.

### 2.8 Multi-sensor information fusion system

The block diagram of the multi-sensor information fusion system performed in this study is shown in Fig 4.

**Fig 4:** Block diagram of the multi-sensor information fusion system.

As shown in Fig 4, this study uses the BPNN and fuzzy control in series to form the multi-sensor information fusion system. The output of the sensor is used as the input of the BPNN, and the output of the BPNN is used as the input of the fuzzy control. This method can greatly amplify the stability of the system.

## 3. Results

### 3.1 Test results of hidden layer nodes

After multiple experiments on Eq (1) above, the test results of hidden layer nodes in this study are shown in Table 1.

**Table 1:** Test results of hidden layer node.

Number of hidden layer nodes	The training steps	Maximum error	Best Validation Performance
6	139	0.0014	0.0013011
7	128	0.0013	0.0005013
8	127	0.0019	0.0027151
9	61	0.0301	0.0035021
10	135	0.0045	0.0020134
11	134	0.0021	0.0030152
12	55	0.0150	0.012131

As shown in Table 1, when the number of hidden nodes is 7, the error of the BPNN is small and the performance is stable. Therefore, this study will select 7 as the number of hidden nodes.

### 3.2 BPNN simulation results

The simulation of BPNN is performed, and the simulation results are shown in Fig 5.

**Fig 5:** BPNN simulation results.

As shown in Fig 5, after 127 iterations, the error of the BPNN reaches the lowest target value, indicating that the BPNN achieves an excellent level of accuracy. The trained BPNN has a running time of 0.0276 s and a mean square error of 0.0013. The smaller the mean square error value is, the higher the accuracy of the BPNN is, which shows that the BPNN meets the high precision requirements of this study.

The detection efficiency of the system is tested, and the test results are shown in Fig 6.

**Fig 6:** BPNN test results.

As shown in Fig 6, the BPNN-based feature layer fusion system can make the most basic judgment of the fire situation. However, the output fire probability value cannot achieve the purpose of judging the fire situation. Therefore, fuzzy control is needed to get a more accurate judgment on fire situations.

### 3.3 Test results of fuzzy control

The simulation of the decision layer is performed, and the test data of the BPNN are input into the decision layer. The processing of the decision layer is shown in Table 2.

**Table 2:** Processing of the decision layer.

Fire probability	Smoldering fire probability	Decision output	Whether the alarm?	Right decision?
0.8166	0.0624	0.532	Yes	Yes
0.9121	0.0443	0.596	Yes	Yes
0.0372	0.8940	0.577	Yes	Yes
0.0631	0.8762	0.531	Yes	Yes
0.0710	0.8543	0.548	Yes	Yes
0.7913	0.0374	0.579	Yes	Yes
0.8104	0.0563	0.566	Yes	Yes

As shown in Table 2, this decision layer control method can make good judgments and decisions on the fire scene conditions. After several tests in this study, they can make accurate judgments on the scene conditions and implement corrective measures. Therefore, this decision layer control method is effective and feasible.

## 4. Discussion

Because of the complex forest environment, flames are easily covered by vegetation such as weeds. Therefore, it is difficult to completely extinguish the fire. At present, most clean up works of remaining fires are undertaken by firefighters. In the jungle with a complex environment, the safety of firefighters is difficult to guarantee. The fires may spread again in the forest at any time, and it is difficult for firefighters to inspect the remaining fires in time and extinguish these fires, resulting in greater losses. Therefore, this study designs a multi-sensor information fusion detection system of the forest remaining fires detection robot, so as to make contributions to the fire protection industry in China.

Through the tests in this study, it is found that when the number of hidden layer nodes of the BPNN is 7, the optimal training result is obtained. On this basis, the test of BPNN in this study is performed. The test results show that after 127 iterations, the error of the BPNN reaches the lowest target value, indicating that the BPNN achieves an excellent level of accuracy. The trained BPNN has a running time of 0.0276 s and a mean square error of 0.0013. The smaller the mean square error value is, the higher the accuracy of the BPNN is, which shows that the BPNN meets the high precision requirements of this study. The BPNN-based feature layer fusion system can make the most basic judgment of the fire situation. However, the output fire probability value cannot achieve the purpose of judging the fire situation. Therefore, fuzzy control is needed to get a more accurate judgment on fire situations. Research and tests of the decision layer show that the multi-sensor fusion detection system designed by this study is effective and highly accurate. Harish et al. (2017) analyzed the fire sensor of the firefighting robot and the pump motor; the fire sensor and the Arduino board were used in the programming of the firefighting agency [21]. The design of the fire sensor above is similar to that in the literature and has achieved consistent results. Aiming to find fire sources, extinguish fire sources, and break the barriers in the forest environment, the firefighting robots designed above combine high-power motor drive control technology, video signal acquisition technology, wireless communication technology, wireless video signal transmission, processing technology, sensor data collection technology, fire source search, and firefighting technology to realize the risks of seriously endangering public safety in emergencies and conduct fire source search based on the wireless remote control and automatic control. Instead of relying solely on rescuers, the designed robots help rescuers get accurate fire field information to minimize the loss of lives and property, as well as reducing the impact on the life and health of firefighters. Tests show that the design scheme of the system is feasible and provides a possible solution for the rescue work of major disasters. The system will have a broad market prospect after production.

The innovation of this study is that in China, there are few pieces of research on forest remaining fires. On this basis, this study provides technical information and theoretical results for subsequent research in this direction, providing materials for the study of forest fire detection technology in China. In addition, this study breaks the traditional method of fire detection and uses robotic detection to greatly reduce labor costs. More importantly, this study reduces the danger of firefighters and ensures the safety of firefighters as much as possible.

## 5. Conclusion

In this study, the BPNN-based forest remaining fires detection method has achieved the expected results. The detection of forest remaining fires is more efficient and robust. The remaining fire may spread again in the forest at any time, making it difficult for firefighters to inspect the fire and ensure timely fire extinguishment, resulting in greater losses. Therefore, the multi-sensor information fusion detection system of firefighting robots is explored. Through this system, robots can help firefighters to inspect fire sites and relieve the disaster, thereby reducing the losses caused by forest fires. Globally, forest fires are frequent in countries with large areas of forests, such as Brazil and Australia. The research on robots for forest fire inspection is also applicable to these countries, helping them achieve the purpose of detecting forest remaining fires. Although this study has achieved some results, there are still some shortcomings in the research process. (1) The research carried out in this study is based on the detection of forest remaining fires. The scenario and its utilization are somehow single. In the future, it will be studied in depth by extending the results of this study to fire detection in densely populated places, such as shopping malls; therefore, the robot can be applied to a variety of different places. (2) The results of this study need further research and analysis. At present, since this study is still in the simulation stage, for complex practical situations, such as forest remaining fire detection under the environmental impact of high-temperature, further research is needed.

## Supporting information

S1 Data (XLS)
